# Meta-Analysis of the Effects of Recombinant Human Brain Natriuretic Peptides on Left Ventricular Remodeling in Patients with Acute Myocardial Infarction

This article has been retracted.

**DOI:** 10.1155/2022/8916791

**Published:** 2022-08-18

**Authors:** Ping Zhu

**Affiliations:** Department of Emergency Medicine, People's Hospital of Daxing District, Beijing, China

## Abstract

**Objective:**

Systematic evaluation of the efficacy of natriuretic recombination in human brain on disease myocardial infarction, left ventricular heart failure, and the efficacy and safety of long-term left ventricular remodeling.

**Methods:**

Computerized search of CNKI, Wanfang database, Wipro Chinese Technology Publications (VIP) numerical database, Chinese Biomedical Literature Database (CBM), Medline Cochrane Library, clinical Trail.Gov clinical collection, and other documents. Randomized controlled trials (RCT) of recombinant human brain natriuretic peptide in the treatment of acute myocardial infarction from inception to December 2021 were searched. Based on the Jadad scale, inclusion-exclusion data for diseases were collected and elaborated by meta by RevMan 5.3 simulation software. In a total of 23 randomized controlled trials, 2 024 cases were used as the basic data, the control group was routinely treated for 1 012 cases, and 1 012 cases in the experimental group were also treated with natriuretic peptide in the recombinant human brain on the previous basis.

**Results:**

In terms of overall efficacy, the experimental group was better than the control group, statistically significant (OR = 4.30, 95% CI (3.26, 5.67), *P* < 0.000 01), left ventricular ejection fraction in the experimental group than the control group (OR = 1.58, 95% CI (1.27, 1.90), *P* < 0.000 01). In terms of a myocardial strain in the left ventricle, the experimental group was superior to the control group. The difference was significant (OR = −0.91, 95% CI (-1.50, -0.33), *P* = 0.002). In terms of the cardiac output volume, the experimental group was superior to the control group (OR = 1.24, 95% CI (0.55, 1.94), *P* = 0.0005). Regarding brain natriuretic peptide precursors, the experimental group was superior to the control group (OR = −4.37, 95% CI (-6.21, -3.25), *P* < 0.00001). In terms of the heart rate, the experimental group was superior to the control group. Measurement of differential significance is as follows: OR = −13.70, 95% CI (-14.95, -12.46), *P* < 0.00001. In terms of contraction, the experimental group was superior to the comparison group (OR = −12.38, 95% CI (-17.98, -6.79), *P* < 0.00001). The experimental group outperformed the control group (OR = −7.42, 95% CI (-8.53, -6.30), *P* < 0.00001). In terms of bad influence, the measurement is as follows: OR = 0.95, 95% CI (0.29, 3.16), *P* = 0.94.

**Conclusion:**

In patients with acute myocardial infarction and left ventricular remodeling, if treated with a heavy treatment of the group of cerebral natriuretic peptide mode, it can increase clinical treatment, improve the cardiac effect, inhibit ventricular remodeling, improve blood pressure and heart rhythm, and have greater clinical treatment and safety.

## 1. Introduction

Acute myocardial infarction is a harmful and clinical life-threatening cardiovascular disease characterized by multimorbidity and high mortality. It mainly shows chest tightness, chest pain, panic, and other symptoms. When an acute myocardial infarction occurs, heart failure often accompanies it. Clinical data show that approximately 8.7% when acute MI occurs develop heart failure. When both diseases occur simultaneously, the 5-year case fatality rate is as high as 55% and increases every year. Heart failure usually causes ventricular filling and impaired ejection [1]. Most current treatments are diuretics, vasodilation, and myocardial reconstruction.

The natriuretic peptide family consists of three biologically active peptides: atrial natriuretic peptide (ANP), brain (or B-type) natriuretic peptide (BNP), and C-type natriuretic peptide (CNP). BNP is a natural antagonist of RAAS, with functions such as catheterization, sodium dilation, vasodilation, inhibition of myocardial fibre hyperplasia, and improvement of myocardial ischemia and hypoxia [2]. However, when an AMI is generated, the amount of BNP excretion is reduced, and it cannot effectively combat the overactivated intraneural excretion system in the body. The group of human brain natriuretic peptides is attributed to endogenous polypeptides, which can antagonize the intraneural excretion system, diuretic and excretion, diffusion of blood vessels, extend cardiac remodeling, and other functions. It can increase the deficiency of BNP in the body, adjust the neuroendocrine system, and rise to the goal of guarding the heart. Recombinant human brain natriuretic peptide (rhBNP) is a new drug for heart failure, with the same functional mechanism as BNP, and has been transformed into the first drug for heart failure in Western developed countries. China has also included the drug in the list of therapeutic drugs. Its function is important for improving cardiac efficacy, such as diuresis, sodium excretion, blood diffusion, constraints on myocardial reconstitution, aldosterone and endothelin excretion, and antisympathetic nervous system. It cannot lead to abnormal heart rate abnormalities. Now, the efficacy and stability of heavy human brain natriuretic peptides for acute myocardial infarction and heart failure need to be completed.

This study traced the correlation from the library establishment to the current RCT, in which the treatment and stability have been systematically evaluated [3]. The significance of this study was to show the role of group of cerebral natriuretic peptide mode in the treatment of acute myocardial infarction and left ventricular, which will present future light for patients. A flow chart of the study is shown in Figure 1.

## 2. Materials and Methods

### 2.1. Diagnostic Criteria

Inclusion criteria are as follows: (1) literature category: randomized controlled clinical trial (RCT). (2) Study number: confirmed acute myocardial infarction (AMI). (3) Intervention method: control group: general routine treatment of Western medicine, covering acute thrombolytic therapy or interventional treatment of respiratory oxygen, diuretic, anticoagulant, antiheart rate abnormalities, antiplatelet aggregation, improved myocardial ischemia, myocardial herb, etc.; treatment group: commonly used treatment of Western medicine+recombinant human brain natriuretic peptide, first give load static push (5 gg/kg), continue 0.0075 g kg^−1^ min^−1^ intravenous drops for 72 h. (4) Results survey: shared efficacy, left ventricular stretching internal diameter (LVDd), left ventricular ejection fraction (LVEF), cerebral natriuretic peptide precursor (NT-ProBNP), cardiac rhythm (HR), compression pressure (SBP), stretching pressure (DBP), etc. Clear specification: (1) unreasonable research and planning and nonrandomized comparative clinical trials; (2) animal trials, review, multiple experiments, and data analysis; and (3) repeatedly cited literature works.

### 2.2. Methods of Searching the Literature

Computers date from this value library to December 2021 and were collected in the published literature from CNKI, WWF, VIP, CBM, PubMed, Cochrane, etc. Search for keywords such as “Recombinant human brain natriuretic peptide,” “acute myocardial infarction,” “heart failure,” and “for left cavity reconstruction” [4].

### 2.3. Specification for Literature Selection and Quality Assessment

Two researchers were randomly selected to search, who removed substandard articles as required and collected literature that met the criteria. Qualified articles were randomly aligned and then evaluated according to the Jadad scoring criteria. Furthermore, the assessment was performed according to the Cochrane bias hazard assessment too, divided by risk [5]. Selection and quality assessment of the literature for the two working staff was done independently without interference from each other. If presented differently, it was assessed by a third-panel member.

### 2.4. Numerical Extraction

Data content: number of diseases, interference method, sample size, clinical efficacy, left ventricular ejection fraction (LVEF), end-diastolic diameter of the left ventricular (LVDd), cerebral natriuretic peptide precursor (NT-ProBNP), cardiac rhythm (HR), systolic blood pressure (SBP), diastolic blood pressure (DBP), and basic information on adverse reactions [6].

### 2.5. Statistical Processing

All statistical calculations were carried out using SPSS statistical software: count data ratio (OR), the weighted average difference (WMD), and 95% confidence interval (CI). The RevMan5.3 software is often used for scientific analysis. Check the heterogeneity of the document and use *I*^2^ to assess its size. If *I*^2^ > 50% showed greater heterogeneity between studies, the meta-analysis used a random effects model [7]. If *I*^2^ was <50%, with less heterogeneity between the studies, a fixed effects model was used for the meta-analysis [8] The observations were stable by excluding the included studies for sensitivity analysis one by one. If the number of documents included in the main indicators is ≥10, the bias can be analyzed by inverted funnel plots [9]. *P* values < 0.05 were considered significant.

## 3. Results

### 3.1. Literature Search Results

Initial screening effect: 67 articles in the Wanfang database, 44 articles in Weipu, CNKI143 articles, and CBM30 articles. After evaluating the retrieved literature, 30 Wanfang articles, Weipu 22 articles, CNKI20 articles, and CBM15 articles were deleted [10]. The remaining 97 articles were integrated, similar 67 articles were removed, 30 articles were classified, and 30 articles were intensively read in full text. There were 23 articles and 2024 cases [11].

### 3.2. Give Quality Evaluation

There are a total of 23 articles, 2024 case No. The 23 articles included in the Jadad score were all 1 to 3, and the overall reassessment was different. All literature reported machine tools and 4 numerical tables, 2 reported computer characteristics, not detailed on-demand scheduling and not blinded in the literature; the whole literature did not report whether scheduling can be performed and hidden [12]; literature did not report the number of people and reasons for departure. The basic characteristics of the study and pursuit are included in Table 1.

### 3.3. Study Quality Evaluation Was Included

It was assessed in the following aspects: (1) random steps: in this study, 23 discussions appeared “randomized”, and 6 studies used the correct randomization method (“computer” method and “table randomization” method). The remaining studies did not mention specific randomized methods and were defined as “unknown risk.” (2) Allocation concealment: none of the 23 studies was discussed and was defined as “unknown risk.” (3) Subject blind method and result evaluator blind: not mentioned in this study and defined as “unknown risk” [13].

### 3.4. Meta-Analysis: 1,666 Cases Were Reported

1. Comparative status of common efficacy after treatment 19 items classified into the literature heterogeneity is *I*^2^ = 0%, clarifying the absence of heterogeneity and elaborating with a firm effect mold. Results: the experimental group is better than the control group in total effective rate. The difference is statistically significant (OR = 4.30, 95% CI (3.26, 5.67), *P* < 0.000 01, *Z* = 10.30) (see Figure 2)
2. Better, the difference has statistical implications. Improved LVEF status after treatment 17 items classified as LVEF status, 1380 cases, heterogeneity testing effect *I*^2^ = 84%. To clarify the heterogeneity, with a smooth effect mold to elaborate. Results: in the case of LVEF improvement, the test group was better and the difference has statistical significance (OR = 1.55, 95% CI (0.74, 1.78), *P* < 0.00001, *Z* = 9.81) (see Figure 3)
3. Improving LVDd status after treatment 8 items were reported in the literature, with a total of 778 cases. Heterogeneity check results *I*^2^ = 93%, elucidating heterogeneity, illustrated with a machine effect mold [13]. Results: under LVDd improvement, the experimental group was better, and the difference had a total statistical academic meaning (OR = −0.91, 95% CI (-1.50, - 0.33), *P* = 0.002, *Z* = 3.04) (see Figure 4)
4. Improved CO status after treatment 4 items were included in the literature to report improved CO status, a total of 350 cases. Heterogenous test *I*^2^ = 89%, elucidating heterogeneity, illustrated by a smooth effect model [14]. Effect: under coimprovement, the experimental group was better, and the difference had a total academic meaning (OR = 1.24, 95% CI (0.55, 1.94), *P* ≤ 0.0015, *Z* = 3.49) (see Figure 5)
5. The literature on improved NT-ProENP status after treatment included 13 Nl-ProBNP status improved in 1 194 cases with heterogeneity examination effect *I*^2^ = 98%, clarifying that the experimental group was better under NP improvement conditions, with total academic significance (OR = −4.37, 95% CI (-5.21, -3.25), *P* < 0.000 01, *Z* = 6.26)
6. Twelve items were included in the literature on improved rhythm status after treatment, reporting rhythm status improvement, totaling 1 016 cases. Heterogeneity trial effect performance *I*^2^ = 0% indicating no heterogeneity, analyzed with a fixed effects model. Results: the test group was more effective in improving heart rate than the control group, and the difference had total academic significance (OR = −13.70, 95% confidence interval (-14.95, -12.46), *P* < 0.00001, *Z* = 2162)
7. Improved SBP status after treatment 9 items were reported in the literature, with a total of 680 cases. Heterogeneity inspection effect performance *I*^2^ = 91%, elucidating heterogeneity, with the random effects mold elaborated. Results: under the condition of SBP improvement, the experimental group is better and different (OR = −12 38, 95% CI (-1798, -679), *P* < 0.00001, *Z* = 434); 248 improved DBP status after treatment 6 subsumed in the literature
8. Improving DBP condition after treatment 6 items included in the literature reported improved DBP, 460 cases. The heterogeneity test results showed *I*^2^ = 0%, indicating no heterogeneity, analyzed with a fixed effects model. Results: the test group was better in improving DBP than the control group and was statistically significant (OR = −7.42, 95% CI (-8.53, -6.30), *P* < 0.000 01, *Z* = 13.03)
9. Adverse reactions: seven adverse reactions reported the occurrence of adverse reactions during the treatment of recombinant human brain natriuretic peptide. The main adverse reactions were the following: hypotension, dizziness, headache, nausea, and palpitations; symptoms can be relieved after adjusted medication speed or withdrawal, and no serious cardiovascular events occurred. The heterogeneity was *I*^2^ = 63%, indicating a heterogeneity, and was analyzed using a random effects model. Results: in terms of adverse reactions, there was no significant difference (OR = 0.95, 95% CI (0.29,3.16), *P* = 0.94, *Z* = 0.08), indicating the safe clinical application of recombinant human brain natriuretic peptide

The sensitivity analysis was performed according to the total effective rate and LVEF of acute myocardial infarction, and the improvement of NT-ProBNP was expounded one by one. The results showed that the removal of random literature did not have any effect on the results, indicating that the results were stable [15].

### 3.5. Sensitivity Elaboration

In view of recombinant human brain natriuretic peptide in the treatment of morbid myocardial apnea, the combined efficacy of weak energy, LVEF, and NT-ProBNP in improving the state was expounded one by one, the effect performance column is elaborated, the effect is removed without a trace of any document, and the reminder effect is stable [16].

### 3.6. Publish-Biased Evaluations

Taking the normative deviation of OR as the vertical axis and OR as the horizontal axis, the common effects of the clinical therapy are drawn to draw a total efficiency funnel plot, and the performance is not completely consistent before and after. It displayed that left and right symmetry is not complete and all consistent, indicating that there may be publication bias (see Figure 6).

When the two groups left the hospital, the difference in the left ventricular poststretch volume (LVEDV) had no obvious meaning (*P* > 0.05), while the rhBNP group had EF values and Tei [17]. The index was significantly higher in the comparison group (*P* < 0.05); 6 months after leaving the hospital, the rhBNP group had a Tei index, EF [17]. The value comparison group still significantly increased (*P* < 0.05), while the rhBNP group's LVEDV and △ LVEDV% were compared to the lower coefficient group, and the difference has a total academic significance (*P* < 0.05).

## 4. Discussion

During periods of acute heart failure or severe heart failure, the inhibitory differential effect of the type of sodium diuretic peptide BNP and circulating neurohormones was unbalanced, although the endogenous BNP level was significantly higher. However, there is still a significant increase in water sodium retention and ventricular filling pressure, manifested in the renin-angiotensin-aldosterone RAAS system into a priming form, endogenous. Through the system of excessive stimulation, resistance or extension of the system circulation, and renal vascular contraction with its precardiac load growth and renal sodium retention, reduce pulmonary capillary wedge pressure, increase sodium secretion, the same period fell low left heart before and after the load, and increase the cardiac index and beat output index [18].

Studies have shown that 1 h after acute myocardial apnea (AMI), endogenous plasma BNP levels rise to 60-fold normal and are initial 24 h sped up to the peak. It can compare the level of ventricular overload at that time of the emotional response. If the area of infarction reaches a certain level, the ventricular tightening effect drops rapidly, and the amount of blood in the heart drops and appears acute heart failure (AHF) [19]. This study shows that after PCI of anterior myocardial apnea in the prewall of disease, the diseased energy is exhausted, and rhBNP or nitroglycerin, nitrous sodium, and other resistance heart power are given. After the treatment of depleted medicinal herbs, plasma renin, angiotensin, and aldosterone water fell evenly compared with before the treatment, but the three neurosecretion hormones in the rhBNP group fell more obviously. This study elucidates that rhBNP is more effective and rapid in treating sick myocardial apnea and adversity. Therefore, the approximate mechanism is speculated to be the exogenous addition of rhBNP in the acute phase of AMI merger disorders [20]. It can better antagonize the transfer stimulation of the neuronal excretory system and can more rapidly alleviate the clinical symptoms of acute heart failure.

Clinical routine EF values are often overestimated because acute myocardial infarction may be a combination of mechanical complications such as heart valve insufficiency, and the cardiac efficacy of such diseases is often overestimated, while the Tei index is not affected by multiple factors such as cardiac sound transmission conditions, heart rhythm, valve conditions, and successive loads. It has a greater correspondence with the pulmonary capillary wedge, so it can effectively and accurately assess cardiac efficacy [21]. This study observed the Tei index and EF at the time of the rhBNP group and 6 months of absence. The values were still significantly higher than in the comparison group (*P* < 0.05). However, there was no significant difference in the volume of left ventricular stretching late stage (LVEDV) after leaving the hospital. After 6 months, the rhBNP group's LVEDV and △ LVEDV% had a shallow decline compared to the control group with, which was probably due to the following: (1) rhBNP pass hit the KATP pathway on the mitochondrial membrane of happy muscle cells, stimulate the mitochondrial stress message waterfall in the cell, appear stress cell guard function, increase myocardial anti-ischemia and hypoxia tolerance, and limit the further expansion of the area of the diseased myocardial infarction to ask [22]. (2) RhBNP can rapidly improve the energy goal of coronary main artery blood flow, so that the diameter and blood flow volume of coronary main artery blood vessels increase significantly, the rotational blocking force falls, and the myocardial tissue in the suffocation area obtains a full blood infusion. (3) RhBNP has the function of antagonizing the sympathetic nervous system. RAAS and other neuronal excretion systems over-invigorate the cardiac toxins produced. The development factor is active in the gene water stabilization system and directly restrains the proliferation, decomposition, and gum of myocardial fibroblasts. RhBNP can antagonize sympathetic nervous system. Cardiac toxins are produced by excessive activation of RAAS and other neuronal excretory systems. Developmental factors are active in the gene water-stable system. They directly inhibit the proliferation, decomposition, and gelation of cardiac fibroblasts and integrate and block the process of ventricular remodeling [23].

Because the result of AMI is mainly myocardial asphyxia, which has an abnormal effect on the heart, the blood volume discharged from the heart is decreased, so that the blood supply of the disease is insufficient, and the renin-angiopoietin-based steroid system (RAAS) is excessively activated. The goal of treatment is to reduce the area of myocardial asphyxia, and the important thing is to prevent synchronization. Although the current cardiac intervention technology is extensive and improved, the survival rate of AMI is significantly improved. Exhaustion rates are also significantly higher [2].

In this study, the treatment and stability of recombinant human brain natriuretic peptide in the treatment of morbid myocardial asphyxia and exhaustion were better described, including 23 articles. The most must have entered 23 articles dedicated, and the effect reminds the application of regrouped human brain natriuretic peptide group than Western medicine common practice treatment results is better, especially in the effective energy, LVEF, LVDd, NT-ProBNP, HR, SBP, DBP, etc. In the bad response, the difference between the two groups is not to have total statistical implications, indicating that the medicinal herbs are stable and robust; however, the scope of this study is preserved, and only 6 have been reported in the literature detailed on-demand literature. The selective bias is also more harmful, and the literature does not report the concealed implementation steps of the distribution. The blindness is not reported, which is probably so high that the bias is high. In addition, the literature is all positive effects, probably due to the positive effect. The manuscript is easy to publish, which will lead to promulgation bias.

As mentioned above, this study summarized the effectiveness of the treatment method of recombinant human brain natriuretic peptide on the combination of diseased myocardial infarction and mental exhaustion and did not perceive the obvious bad repercussions. However, there are also limits of this study. The literature included in this study is all Chinese, and the English literature has not been traced. The selection of surviving literature is likely huge, the quality of the literature is low, and the accuracy of the above research effect will probably have an impact. It is proposed to pay attention to the random steps, blinding, and distribution concealment in future clinical seminars and hopes to present relevant clinical studies with multiple central and large samples to verify the effect of this study [24].

## 5. Conclusion

In patients with acute myocardial infarction and left ventricular remodeling, a heavy treatment of the group of cerebral natriuretic peptide mode can improve the cardiac effect, inhibit ventricular remodeling, and improve blood pressure and heart rhythm, thus having greater clinical treatment and safety.

## Figures and Tables

**Figure 1:** Flow chart of the study.

**Figure 2:** Forest diagram of therapeutic effect of recombinant human brain natriuretic peptide.

**Figure 3:** Forest map was compared with LVEF after recombinant human brain natriuretic peptide.

**Figure 4:** LVDd was used to compare forest map with recombinant human brain natriuretic peptide.

**Figure 5:** CO contrast forest map using recombinant human brain natriuretic peptide.

**Figure 6:** Funnel diagram of clinical efficacy.

**Table 1:** Basic characteristics of the included literature.

Into	Number of cases	Male/female	Means of intervention		Jadad scale	Outcome measures
Study	(T/C)	(*O*)	Control group	Treatment group		
Liu Yanan (2013)	40/40	55/25	Conventional treatment in Western medicine	Control group based+recombinant human brain natriuretic peptides	1	②③⑥⑦
Gong Yun (2019)	46/46	53/39	Conventional treatment in Western medicine	Control group based+recombinant human brain natriuretic peptides	1	①②③④⑤ ⑥
Yang Yunxian (2012)	28/28	36/20	Conventional treatment in Western medicine	Control group based+recombinant human brain natriuretic peptides	1	②③
Fu Bao (2019)	45/45	51/39	Conventional treatment in Western medicine	Control group based+recombinant human brain natriuretic peptides	3	①⑤⑨
Sowangsheng (2014)	34/34	38/30	Conventional treatment in Western medicine	Control group based+recombinant human brain natriuretic peptides	1	①②④⑤⑨
Wang Mingjian (2015)	44/44	53/35	Conventional treatment in Western medicine	Control group based+recombinant human brain natriuretic peptides	1	①②⑤⑥⑦ ⑧
Rahun (201 3)	44/44	46/42	Conventional treatment in Western medicine	Control group based+recombinant human brain natriuretic peptides	1	①②⑤⑥⑦⑧
Lv Tielin (2018)	42/42	47/37	Conventional treatment in Western medicine	Control group based+recombinant human brain natriuretic peptides	1	①
Bassan (2013)	44623	46/28	Conventional treatment in Western medicine	Control group based+recombinant human brain natriuretic peptides	1	①②⑤⑥⑦⑧⑨
Ding Fuyun (2015)	29/29	38/20	Conventional treatment in Western medicine	Control group based+recombinant human brain natriuretic peptides	3	①
Chen Jiming (2019)	36/36	35/37	Conventional treatment in Western medicine	Control group based+recombinant human brain natriuretic peptides	1	①
Ge Zhenrong (2015)	24/26	44633	Conventional treatment in Western medicine	Control group based+recombinant human brain natriuretic peptides	1	②③⑤⑥⑦⑨
Wang Fan (2019)	45/45	55 35	Conventional treatment in Western medicine	Control group based+recombinant human brain natriuretic peptides	1	①②③
Tu Xuanqing (2014)	30/28	3820	Conventional treatment in Western medicine	Control group based+recombinant human brain natriuretic peptides	1	①②③⑤
Chen Jinshui (2015)	114/114	164 64	Conventional treatment in Western medicine	Control group based+recombinant human brain natriuretic peptides	1	①②③⑤
Hu Min (2018)	15/15	15 15	Conventional treatment in Western medicine	Control group based+recombinant human brain natriuretic peptides	3	①⑥⑦⑧
All Silver Hime (2017)	40/40	44 36	Conventional treatment in Western medicine	Control group based+recombinant human brain natriuretic peptides	3	①⑥⑦⑧
Wang Guangjun (2017)	41/41	4636	Conventional treatment in Western medicine	Control group based+recombinant human brain natriuretic peptides	1	②③⑤
Gou Yi (2019)	45/45	4/43	Conventional treatment in Western medicine	Control group based+recombinant human brain natriuretic peptides	1	⑥⑦
Wang Xumin (2018)	80/80	113/47	Conventional treatment in Western medicine	Control group based+recombinant human brain natriuretic peptides	3	①②④⑥⑨
Mapletree Hall (2016)	42/42	4836	Conventional treatment in Western medicine	Control group based+recombinant human brain natriuretic peptides	3	①②⑤⑥
Zou Ruixiu (2016)	15/15	1911	Conventional treatment in Western medicine	Control group based+recombinant human brain natriuretic peptides	1	①②④⑨
Chen Yanchun (2019)	46/46	5/35	Conventional treatment in Western medicine	Control group based+recombinant human brain natriuretic peptides	1	①②③⑤
Nini Wang (2014)	50/50	54 46	Conventional treatment in Western medicine	Control group based+recombinant human brain natriuretic peptides	1	①②⑤⑥⑦⑧⑨

Note: (1) shared performance; (2) LVEF; (3) LVDd; (4) CO; (5) NT-ProBNP; (6) HR; (7) SBP; (8) DBP; (9) bad response.

## Data Availability

The data used to support this study is available from the corresponding author upon request.
